The article "catena-Poly[[aqua­(2,2′-bipyridine-κ2 N,N′)copper(II)]-μ-5-nitro­isophthalato-κ3 O 1,O 1′:O 3]" was retracted in 2012. Reason: fabricated or falsified data.

# *catena*-Poly[[aqua­(2,2′-bipyridine-κ^2^ *N*,*N*′)copper(II)]-μ-5-nitro­isophthalato-κ^3^ *O* ^1^,*O* ^1′^:*O* ^3^]

**DOI:** 10.1107/S1600536808035150

**Published:** 2008-11-08

**Authors:** Lujiang Hao, Xia Liu

**Affiliations:** a College of Food and Biological Engineering, Shandong Institute of Light Industry, Jinan 250353, People’s Republic of China; b Maize Research Insitute, Shandong Academy of Agricultural Science, Jinan 250100, People’s Republic of China

## Abstract

In the asymmetric unit of the title compound, [Cu(C_8_H_3_NO_6_)(C_10_H_8_N_2_)(H_2_O)]_*n*_, there are two symmetry-independent one-dimensional coordination polymers related by a non-crystallographic inversion center. Within the polymers, the Cu^II ^atoms, coordinated by the water mol­ecule and the chelating 2,2′-bipyridine ligands, are bridged by 5-nitro­benzene-1,3-dicarboxyl­ate dianions which act as tridentate ligands; the carboxyl­ate groups exhibit monodentate and symmetric bidentate coordination modes. The Cu^II^ atoms show a strongly distorted octa­hedral coordination geometry. In the crystal structure, the two symmetry-independent coordination polymers form another one-dimensional polymeric structure *via* O—H⋯O hydrogen bonds between coordinated water mol­ecules and carboxyl­ate groups.

## Related literature

For the uses of carboxylic acids in materials science, see: Church & Halvorson (1959 ▶), and in biological systems, see: Okabe & Oya (2000 ▶); Kim *et al.* (2001 ▶).

## Experimental

### 

#### Crystal data

[Cu(C_8_H_3_NO_6_)(C_10_H_8_N_2_)(H_2_O)]
*M* *_r_* = 446.85
Monoclinic,
*a* = 10.1326 (10) Å
*b* = 23.263 (3) Å
*c* = 15.6087 (15) Å
β = 97.28 (2)°
*V* = 3649.6 (7) Å^3^
*Z* = 8
Mo *K*α radiation
μ = 1.25 mm^−1^
*T* = 293 (2) K
0.12 × 0.10 × 0.08 mm

#### Data collection

Bruker APEXII CCD area-detector diffractometer
Absorption correction: multi-scan (*SADABS*; Bruker, 2001 ▶) *T*_min_ = 0.865, *T*_max_ = 0.907
18862 measured reflections
6694 independent reflections
5089 reflections with *I* > 2σ(*I*)
*R*_int_ = 0.025

#### Refinement

*R*[*F* ^2^ > 2σ(*F* ^2^)] = 0.042
*wR*(*F* ^2^) = 0.123
*S* = 1.00
6694 reflections
535 parameters
6 restraints
H atoms treated by a mixture of independent and constrained refinement
Δρ_max_ = 0.83 e Å^−3^
Δρ_min_ = −0.40 e Å^−3^

### 

Data collection: *APEX2* (Bruker, 2004 ▶); cell refinement: *SAINT-Plus* (Bruker, 2001 ▶); data reduction: *SAINT-Plus*; program(s) used to solve structure: *SHELXS97* (Sheldrick, 2008 ▶); program(s) used to refine structure: *SHELXL97* (Sheldrick, 2008 ▶); molecular graphics: *SHELXTL* (Sheldrick, 2008 ▶); software used to prepare material for publication: *SHELXTL*.

## Supplementary Material

Crystal structure: contains datablocks global, I. DOI: 10.1107/S1600536808035150/gk2170sup1.cif

Structure factors: contains datablocks I. DOI: 10.1107/S1600536808035150/gk2170Isup2.hkl

Additional supplementary materials:  crystallographic information; 3D view; checkCIF report

The article "catena-Poly[[aqua­(2,2′-bipyridine-κ2 N,N′)copper(II)]-μ-5-nitro­isophthalato-κ3 O 1,O 1′:O 3]" was retracted in 2012. Reason: fabricated or falsified data.

## Figures and Tables

**Table 1:** Hydrogen-bond geometry (Å, °)

*D*—H⋯*A*	*D*—H	H⋯*A*	*D*⋯*A*	*D*—H⋯*A*
O12—H1*W*⋯O2^i^	0.83 (4)	1.98 (2)	2.742 (3)	153 (4)
O1—H4*W*⋯O10^ii^	0.82 (3)	1.95 (2)	2.724 (3)	158 (4)
O12—H2*W*⋯O5	0.82 (4)	2.07 (3)	2.760 (3)	141 (4)
O1—H3*W*⋯O13	0.83 (3)	2.13 (3)	2.778 (3)	135 (4)

Symmetry codes: (i) ; (ii) .

## supplementary crystallographic information

### Comment

In recent years, carboxylic acids have been widely used as polydentate ligands, which can coordinate to transition or rare earth ions yielding complexes with interesting properties that are useful in materials science (Church & Halvorson, 1959) and in biological systems (Okabe & Oya, 2000). For example, Kim *et al.* (2001) focused on the syntheses of transition metal complexes containing benzene carboxylate and rigid aromatic pyridine ligands in order to study their electronic conductivity and magnetic properties. The importance of transition metal dicarboxylate complexes motivated us to pursue synthetic strategies for these compounds, using 5-nitroisophthalic acid as a polydentate ligand. Here we report the synthesis and X-ray crystal structure analysis of the title compound.

The molecular structure of the title compound is shown in Fig. 1. The title compound, [Cu(C_8_H_3_NO_6_)(C_10_H_8_N_2_)(H_2_O)]_n_ is a one-dimensional coordination polymer (Fig. 2). There are two symmetry independent 1D polymers in the crystal. The Cu(II) atom shows a strongly disordered coordination geometry. It is coordinated by two carboxylate groups from two different 5-nitroisophthalate ligands, 2,2'-bipyridyl and water molecule. The carboxylate groups act in a monodentate and bidentate coordination modes.The symmetry independent polymeric chains are linked via O-H···O hydrogen bonds (Table 1).

### Experimental

A mixture of copper dichloride (0.5 mmol), 2,2'-bipyridine (0.5 mmol), and 5-nitroisophthalic acid (0.5 mmol) in H_2_O (8 ml) and ethanol (8 ml) was sealed in a 25 ml Teflon-lined stainless steel autoclave and kept at 413 K for three days. Blue crystals were obtained after cooling to room temperature (yield  27%). Anal. Calc. for C_18_H_13_CuN_3_O_7_: C 48.34, H 2.91, N 10.74%; Found: C 48.30, H 2.84, N 10.69%.

### Refinement

The H atoms of water molecule were located from difference Fourier maps and were refined with distance restraints: d(H–H) = 1.38 (2) Å, d(O–H) = 0.88 (2) Å, and with a fixed *U*_iso_ of 0.080 Å^2^. All other H atoms were placed in calculated positions with a C—H bond distance of 0.93 Å and refined in the riding model approximation with *U*_iso_(H) = 1.2*U*_eq _ of the carrier atom.

The article "catena-Poly[[aqua­(2,2′-bipyridine-κ2 N,N′)copper(II)]-μ-5-nitro­isophthalato-κ3 O 1,O 1′:O 3]" was retracted in 2012. Reason: fabricated or falsified data.

### Crystal data

**Table:**

[Cu(C_8_H_3_NO_6_)(C_10_H_8_N_2_)(H_2_O)]	*F*_000_ = 1816
*M**_r_* = 446.85	*D*_x_ = 1.627 Mg m^−^^3^
Monoclinic, *P*2_1_/*n*	Mo *K*α radiation λ = 0.71073 Å
Hall symbol: -P 2yn	Cell parameters from 6694 reflections
*a* = 10.1326 (10) Å	θ = 1.8–25.5º
*b* = 23.263 (3) Å	µ = 1.25 mm^−^^1^
*c* = 15.6087 (15) Å	*T* = 293 (2) K
β = 97.28 (2)º	Block, blue
*V* = 3649.6 (7) Å^3^	0.12 × 0.10 × 0.08 mm
*Z* = 8	

### Data collection

**Table:**

Bruker APEXII CCD area-detector diffractometer	6694 independent reflections
Radiation source: fine-focus sealed tube	5089 reflections with *I* > 2σ(*I*)
Monochromator: graphite	*R*_int_ = 0.025
*T* = 293(2) K	θ_max_ = 25.5º
φ and ω scans	θ_min_ = 1.8º
Absorption correction: multi-scan(SADABS; Bruker, 2001)	*h* = −12→10
*T*_min_ = 0.865, *T*_max_ = 0.907	*k* = −28→22
18862 measured reflections	*l* = −18→18

### Refinement

**Table:**

Refinement on *F*^2^	Secondary atom site location: difference Fourier map
Least-squares matrix: full	Hydrogen site location: inferred from neighbouring sites
*R*[*F*^2^ > 2σ(*F*^2^)] = 0.042	H atoms treated by a mixture of independent and constrained refinement
*wR*(*F*^2^) = 0.124	*w* = 1/[σ^2^(*F*_o_^2^) + (0.075*P*)^2^ + 2.4671*P*] where *P* = (*F*_o_^2^ + 2*F*_c_^2^)/3
*S* = 1.00	(Δ/σ)_max_ = 0.003
6694 reflections	Δρ_max_ = 0.83 e Å^−^^3^
535 parameters	Δρ_min_ = −0.40 e Å^−^^3^
6 restraints	Extinction correction: none
Primary atom site location: structure-invariant direct methods	

### Special details

**Table:**

Geometry. All e.s.d.'s (except the e.s.d. in the dihedral angle between two l.s. planes) are estimated using the full covariance matrix. The cell e.s.d.'s are taken into account individually in the estimation of e.s.d.'s in distances, angles and torsion angles; correlations between e.s.d.'s in cell parameters are only used when they are defined by crystal symmetry. An approximate (isotropic) treatment of cell e.s.d.'s is used for estimating e.s.d.'s involving l.s. planes.
Refinement. Refinement of *F*^2^ against ALL reflections. The weighted *R*-factor *wR* and goodness of fit *S* are based on *F*^2^, conventional *R*-factors *R* are based on *F*, with *F* set to zero for negative *F*^2^. The threshold expression of *F*^2^ > σ(*F*^2^) is used only for calculating *R*-factors(gt) *etc*. and is not relevant to the choice of reflections for refinement. *R*-factors based on *F*^2^ are statistically about twice as large as those based on *F*, and *R*- factors based on ALL data will be even larger.

The article "catena-Poly[[aqua­(2,2′-bipyridine-κ2 N,N′)copper(II)]-μ-5-nitro­isophthalato-κ3 O 1,O 1′:O 3]" was retracted in 2012. Reason: fabricated or falsified data.

### Fractional atomic coordinates and isotropic or equivalent isotropic displacement parameters (Å^2^)

**Table:**

	*x*	*y*	*z*	*U*_iso_*/*U*_eq_	
Cu1	1.16168 (4)	0.154431 (15)	0.85573 (3)	0.02711 (13)	
Cu2	0.12372 (4)	0.354405 (16)	0.93350 (3)	0.03053 (13)	
C1	1.1959 (4)	0.07213 (16)	1.0079 (2)	0.0457 (9)	
H1	1.2145	0.1048	1.0416	0.055*	
C2	1.2039 (5)	0.0193 (2)	1.0471 (3)	0.0635 (13)	
H2	1.2268	0.0161	1.1065	0.076*	
C3	1.1773 (5)	−0.02890 (18)	0.9970 (3)	0.0634 (13)	
H3	1.1810	−0.0651	1.0224	0.076*	
C4	1.1452 (4)	−0.02334 (16)	0.9089 (3)	0.0481 (10)	
H4	1.1282	−0.0556	0.8741	0.058*	
C5	1.1388 (3)	0.03117 (13)	0.8732 (2)	0.0291 (7)	
C6	1.1072 (3)	0.04138 (13)	0.7785 (2)	0.0266 (7)	
C7	1.0796 (3)	−0.00183 (15)	0.7180 (2)	0.0376 (8)	
H7	1.0788	−0.0401	0.7354	0.045*	
C8	1.0527 (4)	0.01249 (16)	0.6306 (2)	0.0408 (9)	
H8	1.0328	−0.0160	0.5891	0.049*	
C9	1.0562 (4)	0.06932 (16)	0.6068 (2)	0.0415 (9)	
H9	1.0383	0.0800	0.5491	0.050*	
C10	1.0866 (3)	0.11017 (14)	0.6700 (2)	0.0337 (8)	
H10	1.0889	0.1486	0.6536	0.040*	
C11	0.3761 (3)	0.19406 (14)	0.8105 (2)	0.0284 (7)	
C12	0.8756 (3)	0.17568 (14)	0.8380 (2)	0.0286 (7)	
C13	0.7500 (3)	0.20954 (13)	0.80617 (19)	0.0232 (6)	
C14	0.6258 (3)	0.18759 (13)	0.8202 (2)	0.0252 (6)	
H14	0.6213	0.1526	0.8484	0.030*	
C15	0.5081 (3)	0.21767 (13)	0.79223 (19)	0.0228 (6)	
C16	0.5143 (3)	0.27058 (14)	0.7520 (2)	0.0287 (7)	
H16	0.4375	0.2912	0.7332	0.034*	
C17	0.6391 (3)	0.29176 (14)	0.7409 (2)	0.0300 (7)	
C18	0.7573 (3)	0.26273 (13)	0.7665 (2)	0.0268 (7)	
H18	0.8388	0.2784	0.7574	0.032*	
C19	0.0858 (4)	0.43908 (16)	0.7844 (3)	0.0419 (9)	
H19	0.0717	0.4066	0.7497	0.050*	
C20	0.0710 (4)	0.49282 (18)	0.7464 (3)	0.0506 (10)	
H20	0.0493	0.4965	0.6869	0.061*	
C21	0.0891 (4)	0.54045 (17)	0.7982 (3)	0.0530 (11)	
H21	0.0801	0.5770	0.7741	0.064*	
C22	0.1206 (3)	0.53393 (15)	0.8859 (3)	0.0437 (9)	
H22	0.1312	0.5660	0.9217	0.052*	
C23	0.1365 (3)	0.47885 (13)	0.9207 (2)	0.0331 (8)	
C24	0.1701 (3)	0.46692 (14)	1.0141 (2)	0.0312 (7)	
C25	0.1994 (4)	0.50930 (15)	1.0773 (3)	0.0450 (10)	
H25	0.1976	0.5480	1.0620	0.054*	
C26	0.2313 (4)	0.49311 (18)	1.1632 (3)	0.0505 (10)	
H26	0.2502	0.5209	1.2059	0.061*	
C27	0.2346 (4)	0.43618 (19)	1.1844 (3)	0.0502 (10)	
H27	0.2573	0.4245	1.2414	0.060*	
C28	0.2036 (4)	0.39641 (17)	1.1200 (2)	0.0423 (9)	
H28	0.2048	0.3577	1.1348	0.051*	
C29	0.4118 (3)	0.33262 (14)	0.9445 (2)	0.0276 (7)	
C30	0.5355 (3)	0.29913 (13)	0.9800 (2)	0.0245 (7)	
C31	0.6609 (3)	0.31950 (13)	0.9659 (2)	0.0247 (6)	
H31	0.6668	0.3529	0.9339	0.030*	
C32	0.7773 (3)	0.29078 (12)	0.9988 (2)	0.0230 (6)	
C33	0.7701 (3)	0.24090 (13)	1.0462 (2)	0.0281 (7)	
H33	0.8466	0.2213	1.0687	0.034*	
C34	0.6445 (3)	0.22111 (13)	1.0589 (2)	0.0274 (7)	
C35	0.5281 (3)	0.24928 (14)	1.0278 (2)	0.0273 (7)	
H35	0.4461	0.2350	1.0387	0.033*	
C36	0.9110 (3)	0.31370 (13)	0.9804 (2)	0.0265 (7)	
N1	1.1618 (3)	0.07821 (11)	0.92194 (18)	0.0308 (6)	
N2	1.1133 (2)	0.09711 (10)	0.75448 (17)	0.0256 (6)	
N3	0.1197 (3)	0.43222 (12)	0.86995 (18)	0.0310 (6)	
N4	0.1716 (3)	0.41090 (11)	1.03653 (19)	0.0315 (6)	
N5	0.6350 (3)	0.16771 (13)	1.1080 (2)	0.0421 (8)	
N6	0.6481 (4)	0.34942 (14)	0.7038 (2)	0.0526 (9)	
O1	0.0918 (2)	0.30549 (9)	0.81941 (17)	0.0320 (5)	
O2	0.3006 (2)	0.31188 (9)	0.96166 (16)	0.0358 (6)	
O3	0.4241 (3)	0.37683 (12)	0.90419 (19)	0.0532 (7)	
O4	0.9139 (2)	0.35925 (10)	0.93797 (18)	0.0392 (6)	
O5	1.0167 (2)	0.28721 (10)	1.00723 (16)	0.0360 (6)	
O6	0.5265 (3)	0.14511 (15)	1.1064 (3)	0.0852 (13)	
O7	0.7369 (3)	0.14842 (12)	1.1487 (2)	0.0579 (8)	
O8	0.5457 (3)	0.37104 (19)	0.6687 (4)	0.128 (2)	
O9	0.7554 (3)	0.37294 (13)	0.7091 (2)	0.0734 (10)	
O10	0.9862 (2)	0.19817 (9)	0.82626 (16)	0.0328 (5)	
O11	0.8637 (3)	0.12791 (13)	0.8686 (2)	0.0653 (9)	
O12	1.1948 (2)	0.20384 (9)	0.97015 (16)	0.0319 (5)	
O13	0.2693 (2)	0.22031 (10)	0.78406 (16)	0.0369 (6)	
O14	0.3736 (2)	0.14837 (10)	0.85273 (17)	0.0390 (6)	
H1W	1.245 (4)	0.2303 (13)	0.960 (3)	0.080*	
H2W	1.132 (3)	0.2151 (17)	0.994 (3)	0.080*	
H3W	0.157 (3)	0.2969 (18)	0.795 (3)	0.080*	
H4W	0.042 (4)	0.2781 (13)	0.824 (3)	0.080*	

The article "catena-Poly[[aqua­(2,2′-bipyridine-κ2 N,N′)copper(II)]-μ-5-nitro­isophthalato-κ3 O 1,O 1′:O 3]" was retracted in 2012. Reason: fabricated or falsified data.

### Atomic displacement parameters (Å^2^)

**Table:**

	*U*^11^	*U*^22^	*U*^33^	*U*^12^	*U*^13^	*U*^23^
Cu1	0.0215 (2)	0.0234 (2)	0.0363 (2)	0.00148 (15)	0.00314 (16)	0.00163 (15)
Cu2	0.0210 (2)	0.0245 (2)	0.0466 (3)	0.00113 (15)	0.00654 (18)	0.00113 (16)
C1	0.065 (3)	0.041 (2)	0.031 (2)	0.0004 (19)	0.0076 (18)	0.0047 (16)
C2	0.096 (4)	0.060 (3)	0.033 (2)	0.006 (3)	0.007 (2)	0.014 (2)
C3	0.092 (4)	0.040 (2)	0.059 (3)	0.004 (2)	0.012 (3)	0.031 (2)
C4	0.063 (3)	0.0273 (18)	0.053 (3)	−0.0023 (17)	0.005 (2)	0.0101 (16)
C5	0.0230 (16)	0.0246 (16)	0.0396 (19)	−0.0009 (12)	0.0039 (14)	0.0044 (13)
C6	0.0201 (15)	0.0235 (15)	0.0361 (18)	−0.0006 (12)	0.0037 (13)	0.0017 (13)
C7	0.0313 (18)	0.0270 (17)	0.054 (2)	−0.0024 (14)	0.0052 (16)	−0.0048 (16)
C8	0.036 (2)	0.043 (2)	0.042 (2)	−0.0019 (16)	0.0012 (16)	−0.0122 (16)
C9	0.041 (2)	0.048 (2)	0.034 (2)	0.0023 (17)	−0.0006 (16)	−0.0037 (16)
C10	0.0362 (19)	0.0319 (17)	0.0323 (19)	0.0054 (14)	0.0015 (15)	0.0049 (14)
C11	0.0197 (16)	0.0332 (17)	0.0332 (18)	−0.0034 (13)	0.0071 (13)	−0.0116 (14)
C12	0.0172 (16)	0.0347 (18)	0.0332 (18)	0.0028 (13)	0.0008 (13)	0.0056 (14)
C13	0.0147 (14)	0.0287 (16)	0.0257 (16)	0.0017 (12)	0.0008 (12)	0.0000 (12)
C14	0.0219 (16)	0.0261 (15)	0.0283 (16)	−0.0010 (12)	0.0054 (13)	−0.0006 (13)
C15	0.0156 (14)	0.0280 (15)	0.0252 (16)	−0.0013 (12)	0.0041 (12)	−0.0061 (12)
C16	0.0173 (15)	0.0372 (18)	0.0314 (18)	0.0093 (13)	0.0027 (13)	0.0019 (14)
C17	0.0269 (17)	0.0298 (16)	0.0343 (18)	0.0035 (13)	0.0078 (14)	0.0110 (13)
C18	0.0156 (14)	0.0337 (17)	0.0314 (18)	−0.0016 (12)	0.0039 (12)	0.0049 (13)
C19	0.040 (2)	0.040 (2)	0.049 (2)	0.0029 (16)	0.0137 (17)	0.0071 (17)
C20	0.043 (2)	0.058 (3)	0.052 (2)	0.0069 (19)	0.0135 (19)	0.024 (2)
C21	0.040 (2)	0.034 (2)	0.088 (3)	0.0026 (17)	0.021 (2)	0.027 (2)
C22	0.031 (2)	0.0237 (17)	0.078 (3)	0.0018 (14)	0.0160 (19)	0.0050 (18)
C23	0.0160 (15)	0.0232 (16)	0.062 (2)	0.0000 (12)	0.0137 (15)	0.0010 (15)
C24	0.0149 (15)	0.0292 (17)	0.051 (2)	−0.0005 (12)	0.0090 (14)	−0.0043 (15)
C25	0.032 (2)	0.0279 (18)	0.077 (3)	−0.0019 (15)	0.0121 (19)	−0.0106 (18)
C26	0.034 (2)	0.059 (3)	0.058 (3)	−0.0019 (18)	0.0037 (19)	−0.021 (2)
C27	0.039 (2)	0.064 (3)	0.048 (2)	0.0050 (19)	0.0075 (18)	−0.006 (2)
C28	0.037 (2)	0.043 (2)	0.047 (2)	0.0056 (17)	0.0058 (17)	−0.0007 (17)
C29	0.0166 (15)	0.0327 (17)	0.0326 (18)	0.0031 (13)	−0.0002 (13)	−0.0046 (14)
C30	0.0155 (15)	0.0300 (16)	0.0279 (17)	0.0005 (12)	0.0024 (12)	−0.0048 (12)
C31	0.0192 (15)	0.0241 (15)	0.0312 (17)	−0.0012 (12)	0.0053 (12)	−0.0004 (12)
C32	0.0156 (15)	0.0266 (15)	0.0276 (16)	−0.0004 (11)	0.0059 (12)	−0.0043 (12)
C33	0.0187 (15)	0.0345 (17)	0.0305 (18)	0.0020 (13)	0.0017 (13)	0.0005 (13)
C34	0.0216 (16)	0.0316 (16)	0.0288 (17)	−0.0020 (13)	0.0027 (13)	0.0043 (13)
C35	0.0175 (15)	0.0342 (17)	0.0307 (18)	−0.0059 (13)	0.0050 (13)	0.0015 (13)
C36	0.0140 (15)	0.0294 (16)	0.0370 (18)	0.0009 (12)	0.0073 (13)	−0.0085 (14)
N1	0.0305 (15)	0.0280 (14)	0.0347 (16)	−0.0011 (11)	0.0068 (12)	0.0048 (11)
N2	0.0213 (13)	0.0233 (13)	0.0320 (15)	0.0026 (10)	0.0030 (11)	−0.0005 (11)
N3	0.0216 (14)	0.0277 (14)	0.0446 (18)	0.0022 (11)	0.0075 (12)	0.0052 (12)
N4	0.0239 (14)	0.0268 (14)	0.0445 (18)	0.0028 (11)	0.0071 (12)	−0.0015 (12)
N5	0.0325 (17)	0.0448 (18)	0.0488 (19)	−0.0039 (14)	0.0042 (14)	0.0181 (14)
N6	0.044 (2)	0.049 (2)	0.068 (2)	0.0143 (16)	0.0185 (17)	0.0321 (17)
O1	0.0243 (12)	0.0261 (12)	0.0455 (14)	0.0024 (9)	0.0044 (10)	−0.0001 (10)
O2	0.0148 (11)	0.0301 (12)	0.0621 (16)	0.0023 (9)	0.0033 (10)	−0.0029 (11)
O3	0.0327 (14)	0.0511 (17)	0.075 (2)	0.0086 (12)	0.0035 (13)	0.0290 (15)
O4	0.0241 (12)	0.0291 (12)	0.0669 (17)	−0.0021 (9)	0.0153 (12)	0.0085 (11)
O5	0.0157 (11)	0.0366 (12)	0.0564 (16)	0.0029 (9)	0.0072 (10)	−0.0003 (11)
O6	0.0464 (19)	0.086 (2)	0.116 (3)	−0.0290 (17)	−0.0150 (19)	0.065 (2)
O7	0.0401 (16)	0.0511 (17)	0.083 (2)	0.0105 (13)	0.0080 (15)	0.0336 (15)
O8	0.046 (2)	0.117 (3)	0.226 (5)	0.037 (2)	0.036 (3)	0.131 (4)
O9	0.061 (2)	0.0534 (18)	0.102 (3)	−0.0163 (16)	−0.0027 (19)	0.0388 (18)
O10	0.0121 (10)	0.0274 (11)	0.0583 (15)	0.0017 (8)	0.0015 (10)	−0.0021 (10)
O11	0.0313 (15)	0.0648 (19)	0.101 (2)	0.0135 (13)	0.0130 (15)	0.0564 (18)
O12	0.0267 (12)	0.0261 (11)	0.0415 (14)	0.0039 (9)	−0.0003 (10)	−0.0027 (10)
O13	0.0157 (11)	0.0404 (13)	0.0550 (16)	0.0031 (10)	0.0066 (10)	−0.0012 (11)
O14	0.0223 (12)	0.0378 (14)	0.0583 (16)	−0.0027 (10)	0.0103 (11)	0.0048 (11)

The article "catena-Poly[[aqua­(2,2′-bipyridine-κ2 N,N′)copper(II)]-μ-5-nitro­isophthalato-κ3 O 1,O 1′:O 3]" was retracted in 2012. Reason: fabricated or falsified data.

### Geometric parameters (Å, °)

**Table:**

Cu1—O10	2.049 (2)	C19—N3	1.345 (5)
Cu1—N1	2.052 (3)	C19—C20	1.384 (5)
Cu1—N2	2.078 (3)	C19—H19	0.9300
Cu1—O12	2.115 (2)	C20—C21	1.371 (6)
Cu1—O14^i^	2.158 (2)	C20—H20	0.9300
Cu1—O13^i^	2.258 (2)	C21—C22	1.374 (6)
Cu2—O2	2.046 (2)	C21—H21	0.9300
Cu2—N3	2.062 (3)	C22—C23	1.393 (5)
Cu2—N4	2.086 (3)	C22—H22	0.9300
Cu2—O1	2.104 (2)	C23—N3	1.341 (4)
Cu2—O4^ii^	2.139 (2)	C23—C24	1.481 (5)
Cu2—O5^ii^	2.294 (2)	C24—N4	1.349 (4)
C1—N1	1.350 (5)	C24—C25	1.400 (5)
C1—C2	1.372 (6)	C25—C26	1.391 (6)
C1—H1	0.9300	C25—H25	0.9300
C2—C3	1.373 (6)	C26—C27	1.364 (6)
C2—H2	0.9300	C26—H26	0.9300
C3—C4	1.379 (6)	C27—C28	1.373 (6)
C3—H3	0.9300	C27—H27	0.9300
C4—C5	1.383 (5)	C28—N4	1.346 (5)
C4—H4	0.9300	C28—H28	0.9300
C5—N1	1.337 (4)	C29—O3	1.220 (4)
C5—C6	1.491 (5)	C29—O2	1.284 (4)
C6—N2	1.353 (4)	C29—C30	1.520 (4)
C6—C7	1.383 (5)	C30—C35	1.386 (4)
C7—C8	1.398 (5)	C30—C31	1.400 (4)
C7—H7	0.9300	C31—C32	1.395 (4)
C8—C9	1.375 (5)	C31—H31	0.9300
C8—H8	0.9300	C32—C33	1.382 (4)
C9—C10	1.375 (5)	C32—C36	1.518 (4)
C9—H9	0.9300	C33—C34	1.391 (4)
C10—N2	1.347 (4)	C33—H33	0.9300
C10—H10	0.9300	C34—C35	1.383 (4)
C11—O14	1.253 (4)	C34—N5	1.470 (4)
C11—O13	1.265 (4)	C35—H35	0.9300
C11—C15	1.506 (4)	C36—O4	1.252 (4)
C12—O11	1.222 (4)	C36—O5	1.260 (4)
C12—O10	1.271 (4)	N5—O6	1.216 (4)
C12—C13	1.525 (4)	N5—O7	1.226 (4)
C13—C18	1.390 (4)	N6—O9	1.211 (4)
C13—C14	1.401 (4)	N6—O8	1.218 (4)
C14—C15	1.404 (4)	O1—H3W	0.83 (3)
C14—H14	0.9300	O1—H4W	0.82 (3)
C15—C16	1.387 (4)	O4—Cu2^i^	2.139 (2)
C16—C17	1.388 (5)	O5—Cu2^i^	2.294 (2)
C16—H16	0.9300	O12—H1W	0.82 (4)
C17—C18	1.389 (4)	O12—H2W	0.82 (4)
C17—N6	1.468 (4)	O13—Cu1^ii^	2.258 (2)
C18—H18	0.9300	O14—Cu1^ii^	2.158 (2)
			
O10—Cu1—N1	119.16 (10)	N3—C19—C20	122.2 (4)
O10—Cu1—N2	91.92 (10)	N3—C19—H19	118.9
N1—Cu1—N2	79.26 (10)	C20—C19—H19	118.9
O10—Cu1—O12	87.71 (9)	C21—C20—C19	118.5 (4)
N1—Cu1—O12	93.12 (10)	C21—C20—H20	120.7
N2—Cu1—O12	171.06 (10)	C19—C20—H20	120.7
O10—Cu1—O14^i^	149.84 (9)	C20—C21—C22	119.7 (3)
N1—Cu1—O14^i^	90.99 (10)	C20—C21—H21	120.1
N2—Cu1—O14^i^	94.65 (10)	C22—C21—H21	120.1
O12—Cu1—O14^i^	90.11 (10)	C21—C22—C23	119.4 (4)
O10—Cu1—O13^i^	90.66 (9)	C21—C22—H22	120.3
N1—Cu1—O13^i^	150.04 (10)	C23—C22—H22	120.3
N2—Cu1—O13^i^	98.11 (10)	N3—C23—C22	120.9 (4)
O12—Cu1—O13^i^	90.83 (9)	N3—C23—C24	115.2 (3)
O14^i^—Cu1—O13^i^	59.29 (8)	C22—C23—C24	123.8 (3)
O2—Cu2—N3	119.41 (10)	N4—C24—C25	120.2 (3)
O2—Cu2—N4	91.57 (10)	N4—C24—C23	115.5 (3)
N3—Cu2—N4	78.83 (11)	C25—C24—C23	124.3 (3)
O2—Cu2—O1	87.52 (9)	C26—C25—C24	119.4 (4)
N3—Cu2—O1	94.37 (10)	C26—C25—H25	120.3
N4—Cu2—O1	171.62 (10)	C24—C25—H25	120.3
O2—Cu2—O4^ii^	149.99 (9)	C27—C26—C25	119.5 (4)
N3—Cu2—O4^ii^	90.60 (9)	C27—C26—H26	120.3
N4—Cu2—O4^ii^	94.38 (10)	C25—C26—H26	120.3
O1—Cu2—O4^ii^	90.54 (10)	C26—C27—C28	118.7 (4)
O2—Cu2—O5^ii^	91.14 (9)	C26—C27—H27	120.6
N3—Cu2—O5^ii^	149.09 (9)	C28—C27—H27	120.6
N4—Cu2—O5^ii^	96.95 (10)	N4—C28—C27	123.0 (4)
O1—Cu2—O5^ii^	91.40 (9)	N4—C28—H28	118.5
O4^ii^—Cu2—O5^ii^	58.96 (8)	C27—C28—H28	118.5
N1—C1—C2	122.1 (4)	O3—C29—O2	125.0 (3)
N1—C1—H1	119.0	O3—C29—C30	119.1 (3)
C2—C1—H1	119.0	O2—C29—C30	115.9 (3)
C1—C2—C3	118.7 (4)	C35—C30—C31	118.7 (3)
C1—C2—H2	120.6	C35—C30—C29	121.8 (3)
C3—C2—H2	120.6	C31—C30—C29	119.5 (3)
C2—C3—C4	119.7 (4)	C32—C31—C30	121.5 (3)
C2—C3—H3	120.1	C32—C31—H31	119.3
C4—C3—H3	120.1	C30—C31—H31	119.3
C3—C4—C5	118.8 (4)	C33—C32—C31	120.0 (3)
C3—C4—H4	120.6	C33—C32—C36	120.3 (3)
C5—C4—H4	120.6	C31—C32—C36	119.7 (3)
N1—C5—C4	121.7 (3)	C32—C33—C34	117.7 (3)
N1—C5—C6	115.7 (3)	C32—C33—H33	121.1
C4—C5—C6	122.6 (3)	C34—C33—H33	121.1
N2—C6—C7	121.3 (3)	C35—C34—C33	123.2 (3)
N2—C6—C5	114.6 (3)	C35—C34—N5	118.3 (3)
C7—C6—C5	124.1 (3)	C33—C34—N5	118.4 (3)
C6—C7—C8	119.4 (3)	C34—C35—C30	118.9 (3)
C6—C7—H7	120.3	C34—C35—H35	120.5
C8—C7—H7	120.3	C30—C35—H35	120.5
C9—C8—C7	118.9 (3)	O4—C36—O5	121.0 (3)
C9—C8—H8	120.5	O4—C36—C32	118.6 (3)
C7—C8—H8	120.5	O5—C36—C32	120.4 (3)
C8—C9—C10	118.8 (3)	O4—C36—Cu2^i^	57.03 (16)
C8—C9—H9	120.6	O5—C36—Cu2^i^	64.09 (16)
C10—C9—H9	120.6	C32—C36—Cu2^i^	174.0 (2)
N2—C10—C9	123.0 (3)	C5—N1—C1	119.0 (3)
N2—C10—H10	118.5	C5—N1—Cu1	115.6 (2)
C9—C10—H10	118.5	C1—N1—Cu1	125.1 (2)
O14—C11—O13	120.5 (3)	C10—N2—C6	118.5 (3)
O14—C11—C15	119.1 (3)	C10—N2—Cu1	126.8 (2)
O13—C11—C15	120.4 (3)	C6—N2—Cu1	114.8 (2)
O14—C11—Cu1^ii^	58.05 (16)	C23—N3—C19	119.2 (3)
O13—C11—Cu1^ii^	62.60 (17)	C23—N3—Cu2	115.6 (2)
C15—C11—Cu1^ii^	174.8 (2)	C19—N3—Cu2	124.6 (2)
O11—C12—O10	124.3 (3)	C28—N4—C24	119.1 (3)
O11—C12—C13	118.5 (3)	C28—N4—Cu2	126.4 (2)
O10—C12—C13	117.1 (3)	C24—N4—Cu2	114.5 (2)
C18—C13—C14	119.6 (3)	O6—N5—O7	123.5 (3)
C18—C13—C12	121.0 (3)	O6—N5—C34	118.3 (3)
C14—C13—C12	119.4 (3)	O7—N5—C34	118.2 (3)
C13—C14—C15	121.0 (3)	O9—N6—O8	123.4 (3)
C13—C14—H14	119.5	O9—N6—C17	119.1 (3)
C15—C14—H14	119.5	O8—N6—C17	117.6 (4)
C16—C15—C14	119.8 (3)	Cu2—O1—H3W	118 (3)
C16—C15—C11	120.1 (3)	Cu2—O1—H4W	112 (3)
C14—C15—C11	120.0 (3)	H3W—O1—H4W	113 (4)
C15—C16—C17	117.8 (3)	C29—O2—Cu2	122.8 (2)
C15—C16—H16	121.1	C36—O4—Cu2^i^	93.58 (18)
C17—C16—H16	121.1	C36—O5—Cu2^i^	86.30 (19)
C16—C17—C18	123.9 (3)	C12—O10—Cu1	121.3 (2)
C16—C17—N6	118.4 (3)	Cu1—O12—H1W	106 (3)
C18—C17—N6	117.6 (3)	Cu1—O12—H2W	121 (3)
C13—C18—C17	117.9 (3)	H1W—O12—H2W	112 (4)
C13—C18—H18	121.0	C11—O13—Cu1^ii^	87.6 (2)
C17—C18—H18	121.0	C11—O14—Cu1^ii^	92.45 (19)

Symmetry codes: (i) *x*+1, *y*, *z*; (ii) *x*−1, *y*, *z*.

The article "catena-Poly[[aqua­(2,2′-bipyridine-κ2 N,N′)copper(II)]-μ-5-nitro­isophthalato-κ3 O 1,O 1′:O 3]" was retracted in 2012. Reason: fabricated or falsified data.

### Hydrogen-bond geometry (Å, °)

**Table:**

*D*—H···*A*	*D*—H	H···*A*	*D*···*A*	*D*—H···*A*
O12—H1W···O2^i^	0.83 (4)	1.98 (2)	2.742 (3)	153 (4)
O1—H4W···O10^ii^	0.82 (3)	1.95 (2)	2.724 (3)	158 (4)
O12—H2W···O5	0.82 (4)	2.07 (3)	2.760 (3)	141 (4)
O1—H3W···O13	0.83 (3)	2.13 (3)	2.778 (3)	135 (4)

Symmetry codes: (i) *x*+1, *y*, *z*; (ii) *x*−1, *y*, *z*.
